# Effects of delta-opioid receptor agonist pretreatment on the cardiotoxicity of bupivacaine in rats

**DOI:** 10.1186/s12871-022-01568-x

**Published:** 2022-01-12

**Authors:** Chenran Wang, Shen Sun, Jing Jiao, Xinhua Yu, Shaoqiang Huang

**Affiliations:** 1 Department of Anesthesia, Obstetrics & Gynecology Hospital of Fudan University, Shanghai, China; 2 Division of Epidemiology, Biostatistics and Environmental Health, Scholl of Health, University of Memphis, Memphis, USA

**Keywords:** Bupivacaine, Cardiotoxicity, Delta-opioid receptor (DOR), BW373U86, Local anesthetic systemic toxicity (LAST)

## Abstract

**Background:**

Delta-opioid receptor is widely expressed in human and rodent hearts, and has been proved to protect cardiomyocytes against ischemia/reperfusion and heart failure. The antagonist of delta-opioid receptor could block the rescue effect of lipid emulsion against local anesthetic cardiotoxicity. However, no evidence is available for the direct effect of delta-opioid-receptor agonists on the cardiotoxicity of local anesthetics.

**Methods:**

Anesthetized Sprague Dawley rats were divided into five groups. Group NS received 2 ml·kg^−1^·min^−1^ normal saline, group LE received 2 ml·kg^−1^·min^−1^ 30% lipid emulsion and group BW received 0.1, 1.0, or 5.0 mg/kg BW373U86, a delta-opioid-receptor agonist, for 5 min. Then 0.5% bupivacaine was infused intravenously at a rate of 3.0 mg·kg^−1^·min^−1^ until asystole. The time of arrhythmia, 50% mean arterial pressure-, 50% heart rate-reduction and asystole were recorded, and the dose of bupivacaine at each time point was calculated.

**Results:**

All three different doses of BW373U86 did not affect the arrhythmia, 50% mean arterial pressure-reduction, 50% heart rate-reduction and asystole dose of bupivacaine compared with group NS. 30% LE significantly increased the bupivacaine threshold of 50% mean arterial pressure-reduction (17.9 [15.4–20.7] versus 7.2 [5.9–8.7], *p* = 0.018), 50% heart rate-reduction (18.7 ± 4.2 versus 8.8 ± 1.7, *p* < 0.001) and asystole (26.5 [21.0–29.1] versus 11.3 [10.7–13.4], *p* = 0.008) compared with group NS. There was no difference between group LE and group NS in the arrhythmia dose of bupivacaine (9.9 [8.9–11.7] versus 5.6 [4.5–7.0], *p* = 0.060).

**Conclusions:**

Our data show that BW373U86 does not affect the cardiotoxicity of bupivacaine compared with NS control in rats. 30% LE pretreatment protects the myocardium against bupivacaine-induced cardiotoxicity.

## Background

With the development of enhanced recovery after surgery (ERAS) and labor analgesia, peripheral nerve block and epidural anesthesia become more and more important for their indispensable role in comfort medicine. Local anesthetic systemic toxicity (LAST) is the adverse effect of regional anesthesia due to unexpected local anesthetics absorbed or infused into the bloodstream [1]. The main symptoms of LAST are central nervous systemic toxicity and cardiotoxicity, of which cardiotoxicity is life-threatening [2]. Lipid emulsion (LE) has been reported to resuscitate LAST successfully in animal experiments and clinical practices [3, 4]. A widely accepted theory of LE rescue is that lipophilic local anesthetics are absorbed into the lipid phase of plasma from tissues [5]. Thus, the toxicity of local anesthetics to tissue is mitigated by LE. However, in 2015, Partownavid et al. [6] reported that LE fails to rescue rats against bupivacaine-induced cardiotoxicity when a high-dose of delta-opioid receptor (DOR) antagonist was preconditioned. This indicates that DOR is involved in the LE rescue of LAST.

DOR is widely expressed in human and rodent cardiomyocytes. And the expression of DOR increases in response to heart failure, hypoxia, aging, and other physical or pathological stimuli [7]. Many studies have proved that agonists of DOR can protect the myocardium against ischemia/reperfusion and heart failure [8–11]. However, no evidence is available concerning the direct effect of DOR agonists on the cardiotoxicity of local anesthetics.

We hypothesized that the agonist of DOR can protect the heart against bupivacaine-induced cardiotoxicity in rats. The purpose of this study is to investigate whether DOR agonist has protective effects on bupivacaine cardiotoxicity. We pretreated anesthetized Sprague Dawley rats with normal saline, lipid emulsion, and three different doses of BW373U86 (0.1, 1.0, 5.0 mg/kg), a DOR agonist, before bupivacaine infusion. Our primary outcome is the asystole dose of bupivacaine in rats. Our secondary outcomes are the doses of bupivacaine when arrhythmia, 50% mean arterial pressure (MAP)-reduction, and 50% heart rate (HR)-reduction occur.

## Methods

### Animals

The animal study was reviewed and approved by the Animal Care and Use Committee of Fudan University on 16 March 2021 (ethic approval ID: 20,210,316–001) and performed according to the National Institutes of Health Guide for the Care and Use of Laboratory Animals. All animal experiments were reported in compliance with the ARRIVE guidelines. Thirty male Sprague Dawley rats aged 5–6 weeks were purchased from Shanghai JieSiJie Laboratory Animals Co. Ltd (Shanghai, China) and housed in a standard environment (23 ± 1℃, 50% relative humidity and 12-h day/night cycle) for more than 7 days before experiments.

### Anesthesia and Monitoring

This model of LAST has been used by many previous studies [2, 4, 6]. Rats (240–280 g) fasted for 12 h before experiments with free access to water. The animals were anesthetized with 350 mg/kg chloral hydrate intraperitoneally. Then they were nasally ventilated using a rodent animal ventilator (ALC-V8, Shanghai Alcott biotech CO.LTD, Shanghai, China). The ventilator settings are as follows: respiratory rate 60 breaths/min, tidal volume 2 ml/100 g, and inspiratory to expiratory ratio 1:2. Sevoflurane (1–2%) in 30% O_2_ was started before the median incision in the neck was made [12]. The right jugular vein and the left carotid artery were intubated with a silastic tube (external diameter × internal diameter = 1.0 × 0.5 mm). Then, rats were intubated by tracheotomy with a 16G angio-catheter. Last, three electrode needles were inserted subcutaneously in both forelimbs and left hindlimb to measure Electrocardiogram (ECG). ECG and invasive arterial blood pressure were constantly recorded with a monitor. After all invasive procedures were finished, sevoflurane was discontinued, the time of surgery (time from neck incision to the end of invasive procedures) was recorded. Rats were allowed to stabilize for 10-15 min. At the end of the stabilization period, HR and MAP were recorded as baseline values. Rectal temperature was maintained at 37 ± 1℃ by a heater throughout the experiment.

### Experimental Procedures

Thirty rats were randomly assigned to five groups (*n* = 6 for each) according to random numbers. All liquids were infused through the right jugular vein using an infusion pump (B. Braun Medical Co., Ltd, Suzhou, China). Group NS received 2 ml·kg^−1^·min^−1^ normal saline for 5 min; group LE received 2 ml·kg^−1^·min^−1^ 30% lipid emulsion (80PE018, Sino-Swed Pharmaceutical Corp. Ltd, Jiangsu, China) for 5 min; and BW groups received 0.1, 1.0 or 5.0 mg/kg (diluted in 10 ml/kg normal saline) BW373U86 (Cat. No. 1663, Tocris Bioscience, USA) for 5 min. The low, median and high doses of BW373U86 were set as 0.1, 1.0, and 5.0 mg/kg according to the previous study [13–16]. After a 1-min wait, which was the time of changing syringes and resetting the velocity of the infusion pump, 0.5% bupivacaine (090,809, Shanghai Harvest Pharmaceutical CO., LTD, Shanghai, China) at a rate of 3.0 mg·kg^−1^·min^−1^ was started to infuse until asystole occurs. Rats were anesthetized with 350 mg/kg chloral hydrate. Thus, animals went into cardiac arrest gradually under anesthesia at the end of the study.

The following toxic endpoints were recorded by an observer unaware of the grouping, and the doses of bupivacaine at each endpoint were calculated: the first arrhythmia, defined as the appearance of cardiac rhythm disturbance on the ECG accompanied by an abnormal pulsation on the arterial pressure trace; 50% MAP-reduction, defined as the MAP of 50% baseline value; 50% HR-reduction, defined as the HR of 50% baseline value; and asystole, defined as the lack of recognizable beat on the ECG for 10 s after the appearance of the last systole. These observed indexes were decided following previous studies [4, 9, 17].

### Statistical Analysis

The software program of Power and Sample Size (PASS15.0.5, NCSS Inc, Kaysville, UT) was used to calculate the sample size [2]. Based on the preliminary experiments of 0.5% bupivacaine at a rate of 3.0 mg·kg^−1^·min^−1^. The mean asystole doses of group NS, LE, 0.1, 1.0, and 5.0 mg/kg BW are 12.1 25.5 14.4 13.2 12.9, and the standard errors are 2.3 5.0 3.1 4.0 4.0 respectively. Power was set at 0.90; significance was set at 0.05, and one-way analysis of variance (ANOVA) was used. The effect size of 5 was estimated. Considering the loss potential and errors, 6 rats for each group were decided.

Data were analyzed with SPSS (version 20.0; Chicago, Illinois, USA) for Windows by a statistician who is blinded to the grouping. The Shapiro–Wilk test was used to test for normal distribution. Normal-distributed measures and abnormal-distributed measures were presented as mean ± standard deviation and median [interquartile range] respectively. Normally distributed measures were compared using a one-way ANOVA model and abnormally distributed measures were compared using the Kruskal–Wallis test. The individual pairwise mean comparisons were adjusted with the Tukey studentized range criterion or Dunn’s test to account for multiple comparisons. The family-wise significance for all tests is set at *p* < 0.05.

## Results

The timeline of the experiment is shown in Fig. 1. The baseline values of weight, MAP, HR and invasive surgery time are presented in Table 1, and no difference was observed among these five groups.

**Fig. 1:** Timeline of the experiment. At the baseline, rats were infused with 2 ml·kg^−1^··min^−1^ normal saline, 30% lipid emulsion, 0.1, 1.0, or 5.0 mg/kg BW373U86, the agonist of delta-opioid receptor for 5 min. After waiting 1 min to change the syringe and the speed of the infusion pump, 0.5% bupivacaine 3.0 mg·kg^−1^··min^−1^ was started to infuse until asystole occurs

**Table 1:** Baseline values

	NS	LE	0.1 BW	1.0 BW	5.0 BW
Weight (g)	262.8 ± 11.9	262.2 ± 9.0	263.7 ± 9.0	263.7 ± 6.5	262.0 ± 6.5
MAP (mmHg)	78.8 ± 9.9	77.7 ± 10.1	87.5 ± 4.5	77.0 ± 5.7	89.2 ± 14.5
HR (beats/min)	221.6 ± 32.2	225.0 ± 42.2	221.5 ± 20.3	227.3 ± 39.7	217.8 ± 28.5
Surgery time (min)	14.6 ± 1.1	13.0 ± 1.5	13.0 ± 2.0	14.0 ± 0.6	13.8 ± 1.9

Table 1 Baseline values. Values are presented as mean ± standard deviation, *n* = 6 for each group. There was no difference in baseline values among NS, LE, 0.1, 1.0, and 5.0 BW groups. Abbreviations: *NS* normal saline, *LE* lipid emulsion, *BW* BW373U86, the agonist of delta-opioid receptor, *MAP* mean arterial pressure, *HR* heart rate. Surgery time: time from neck incision to the end of all invasive procedures

All three doses of BW373U86 (0.1, 1.0, and 5.0 mg/kg) had no effect on the bupivacaine threshold of arrhythmia, 50% MAP-reduction, 50% HR-reduction, or asystole compared with NS control (Fig. 2). 30% LE increased the bupivacaine threshold of 50% MAP-reduction (17.9 [15.4–20.7] versus 7.2 [5.9–8.7], *p* = 0.018), 50% HR-reduction (18.7 ± 4.2 versus 8.8 ± 1.7, *p* < 0.001) and asystole (26.5 [21.0–29.1] versus 11.3 [10.7–13.4], *p* = 0.008) compared with group NS. There is no difference between group LE and group NS on the arrhythmia dose of bupivacaine (9.9 [8.9–11.7] versus 5.6 [4.5–7.0], *p* = 0.060).

**Fig. 2:** The bupivacaine threshold of different cardiotoxic endpoints: **a** arrhythmia; **b** 50% MAP-reduction; **c** 50% HR-reduction; **d** asystole. Differences were found between group NS and LE in the bupivacaine dose of 50% MAP-reduction, 50% HR-reduction, and asystole. Abbreviations: *NS* normal saline, *LE* lipid emulsion, *BW* BW373U86, the agonist of delta-opioid receptor, *MAP* mean arterial pressure, *HR* heart rate.^*^p < 0.05, ^**^p < 0.01, ^***^p < 0.001

## Discussion

The cardioprotective effects of DOR in ischemia/reperfusion and heart failure have long been highlighted in both in vivo and in vitro studies [8, 10, 18, 19], while the effect of DOR agonist on the cardiotoxicity of local anesthetics has never been explored before. Our study firstly investigated the effect of DOR agonist on the cardiotoxicity of bupivacaine in rats, however, we didn’t observe any positive effect.

DOR is widely expressed in human and rodent myocardium and has been proved to involve in the cardioprotective and neuroprotective procedures in myocardial ischemia/reperfusion [8, 9, 13, 19, 20]. The mechanisms of DOR protective effects on the myocardium include triggering PKC, ERK1/2, Akt/PIK3, and other pathways. These activated pathways may confer protection through regulating anti-apoptotic and autophagy elements, releasing NO, inhibiting Ca^2+^ overload, phosphorylating GSK3β, inhibiting mitochondrial permeability transition pore (mPTP) open [21], and activating mitochondrial K_ATP_ [7, 22], of which mitochondrial function is closely involved. Both Furado et al. [21] and Bell et al. [19] reported that the contraction of human atrial trabeculae after ischemia/reperfusion is significantly increased with Delta 2 opioid D-Ala2-Leu5 enkephalin (DADLE, a DOR agonist) treatment. And the protective effect of DADLE is mediated by both the mPTP opener and mitochondrial K_ATP_ channel (mK_ATP_).

It has been proved that bupivacaine exerts an adverse effect on the myocardium by inhibiting ion channels open (including sodium, potassium, and calcium channels) and disturbing mitochondrial energy metabolism [23, 24]. Chen Y et al. [25] reported that ropivacaine injuries human neuron SH-5Y5Y through opening mPTP, decreasing ATP production and inducing other mitochondrial dysfunctions. Thus, we hypothesized that DOR may protect the myocardium against bupivacaine by modulating mitochondrial function. However, we didn’t observe any protective effects of DOR on the cardiotoxicity of bupivacaine in rats.

We chose 0.1, 1.0, and 5.0 mg/kg BW373U86, which is the low, median, and high doses of BW that have been proved to activate DOR in rats [13–16]. Therefore, we think it’s sufficient to conclude that BW does not affect the cardiotoxicity of bupivacaine. This result seems contradictory to that of Partownavid et al. [6]. Partownavid et al. reported that DOR antagonists can abolish the therapeutic effect of LE against bupivacaine toxicity, which indicates that LE may exert protective effects by activating DOR. The reason for the difference may be due to the complex mechanism of LE rescuing LAST. DOR may only play an important role in it. However, it’s not enough to ameliorate the toxicity of local anesthetics by activating DOR alone.

Unlike the 20% LE that is used mostly, we used 30% LE. Because 30% LE has been proved to exert cardioprotective effects against LAST as well [4], and the ratio of the main effective ingredients of 30% LE to that of 20% LE is 2:3. Thus we chose 2 ml·kg^−1^·min^−1^ 30% LE following the dose of LE used by Weinberg and other researchers [4, 26, 27].

The median doses of bupivacaine producing asystole in group NS and group LE of our study are 11.3 mg/kg and 26.5 mg/kg respectively. Both the two doses are lower than that of the study of Weinberg (group NS 17.7 mg/kg and group LE 49.7 mg/kg) [4]. We think this is mainly because we discontinued sevoflurane while Weinberg et al. did not. And inhale anesthetics, like sevoflurane and isoflurane, can prolong the death time of local anesthetics [28, 29]. Because inhale anesthetics exert cardioprotective effects against LAST, thus we stopped sevoflurane as soon as finishing the invasive procedure and waited for 10–15 min to allow rats to exhale sevoflurane so that the result is more credible.

There are some limitations of our study. First, we just observed a phenomenon. This is mainly because the negative outcome limits further investigations on the mechanism. Second, we only studied the preventative effect without the resuscitative effect of DOR agonist on LAST. For lipid emulsion has been considered as the golden standard for the rescue of LAST, and we aimed to look for one drug that may help to prevent the cardiotoxicity of local anesthetics. Third, we didn’t mirror expired CO_2_ concentration in this experiment, which may affect cardiac function. However, most of the literature we referred didn’t mirror expired CO_2_ concentration, too. And the ventilator settings of our experiment are the same as those of others.

## Conclusions

Our study demonstrates that BW373U86 does not affect the cardiotoxicity of bupivacaine in rats compared with normal saline control. 30% lipid emulsion can protect the myocardium against bupivacaine-induced cardiotoxicity.

## Data Availability

The datasets used and/or analyzed during the current study are available from the corresponding author on reasonable request.

## Abbreviations

NS: Normal saline
LE: Lipid emulsion
BW: BW373U86
ERAS: Enhanced recovery after surgery
MAP: Mean arterial pressure
HR: Heart rate
LAST: Local anesthetic systemic toxicity
ECG: Electrocardiogram
DADLE: Delta 2 opioid D-Ala2-Leu5 enkephalin
mPTP: mitochondrial permeability transition pore
